# The Association between Long Noncoding RNA over Expression and Poor Prognosis of Liver Cancer: A Meta-Analysis

This article has been retracted.

**DOI:** 10.1155/2021/1395131

**Published:** 2021-11-24

**Authors:** Leiqing Wang, Junzhi Sheng, Haojie Zhang, Baoyuan Xie, Linbiao Xiang, Dong Liu, Xinyuan Zhang, Peihao Zhang, Jinjin Liu

**Affiliations:** ^1^The First School of Clinical Medicine of Lanzhou University, Lanzhou 730000, Gansu, China; ^2^Department of Clinical Medicine, Medical College, Wuhan University of Science and Technology, Wuhan 430065, Hubei, China; ^3^The Second School of Clinical Medicine of Lanzhou University, Lanzhou 730000, Gansu, China; ^4^The School of Clinical Medicine of Shi Hezi University, Shi Hezi 832000, Xinjiang, China; ^5^The School of Clinical Medicine of Weifang Medical University, Weifang 261000, Shandong, China; ^6^Department of Endocrinology, The First Hospital of Lanzhou University, No. 1 West Donggang Road, Lanzhou, Gansu 730000, China

## Abstract

**Background:**

Long noncoding RNA (lncRNA) is considered to be a mediator of carcinogenesis, which may be associated with liver cancer survival. However, the relationship remains inconclusive. Meta-analysis was conducted to analytically review the association between the lncRNA expression level and clinicopathological characteristics and prognostic value of hepatic carcinoma.

**Materials and Methods:**

Four databases including Embase, PubMed, Web of Science, and the Cochrane Library were searched to collect studies about the relation between lncRNA overexpression and prognosis of liver cancer, dating from the earliest records of these databases to March 2021. Two researchers independently screened the data and literature to perform a stringent evaluation of the quality of material involved in the study. Meta-analysis was performed by Stata 16.0 software on 42 case-control studies with 6293 samples.

**Results:**

The outcomes of meta-analysis are presented as follows: lncRNA overexpression patients had later TNM stage (OR = 0.36, 95% CI (0.31, 0.41), *P* < 0.001), lower histological grade (OR = 0.56, 95%CI (0.49, 0.65), *P* < 0.001), more vascular invasion (OR = 2.02, 95% CI (1.74, 2.35), *P* < 0.001), bigger tumor size (OR = 2.28, 95% CI (2.00, 2.60), *P* < 0.001), more severe liver cirrhosis (OR = 1.39, 95% CI(0.1.16, 1.66), *P* < 0.001), more likely to metastasize (OR = 1.80, 95%CI(1.49, 2.18), *P* < 0.001), and more tumor numbers (OR = 0.72, 95% CI (0.62, 0.84), *P* < 0.05). lncRNA over expression patients had shorter OS (HR = 2.32, 95 CI% (2.08, 2.59), *P* < 0.01, RFS (HR = 2.19, 95 CI% (1.72, 2.78), *P* < 0.01), and DFS (HR = 2.01, 95 CI% (1.57, 2.57), *P* < 0.01).

**Conclusions:**

Overexposure of lncRNA is a poor prognostic feature for patients with hepatic carcinoma. The scope of our study was limited because of a lack of relevant research and the poor representativeness and varying quality of the studies involved in the current meta-analysis. Our conclusion still requires higher studies for further validation. This trial is clinically registered with CRD4201920620.

## 1. Introduction

Hepatic carcinoma is one of the most commonly occurring malignant cancers, with morbidity and mortality ranked sixth and second, respectively, causing serious threats to human health [1, 2]. According to statistics in 2012, there are about 780,000 novel patients reported and 740,000 deaths across the globe. The incidence of China accounts for 50%, and it shows an upward trend [3]. So far, it is believed that genetic and environmental factors, both cause tumorigenesis, but the specific pathogenesis of liver cancer has not been completely clarified. Currently, surgical treatment is still the most effective and radically curable method, but a considerable number of patients with liver cancer cannot be suffered from surgery or have lost the best time for surgery. Therefore, it is urgently necessary to find new effective markers that are specifically expressed in hepatic malignant to improve the diagnosis and the accuracy of judgment on prognosis. Over the last few years, the function of long noncoding RNA (lncRNA) in many pathological and physiological pathways has been gradually explored, and it is also aberrantly expressed in some malignant tumors, regulating the spread, variation, and metastasis of cancerous cells [4].

lncRNA is a kind of endogenic RNA 200 or more nucleotides long, which is extensively present in *Homo sapiens*. It has no protein-coding function and lacks a specific open reading frame (ORF) [5], which was considered to be a nonsignificant byproduct of transcription in the early stage [6–8]. Over the years, due to the advancement of high-resolution chips and high-throughput sequencing technologies, the research on transcriptome regulation has been increasingly deepened, and it is found that lncRNA not only plays a significant role in transcriptional interference but also in the process of some histological development, tumorigenesis, and tumor metastasis [9–11]. Researchers have found that aberrant expression of lncRNA affects the prognosis of liver cancer, associated with metastasis, TNM stage, and other clinicopathological characteristics of liver cancer [12]. Therefore, lncRNA could be a novel marker for the diagnosis, prognosis of liver cancer, and a possible therapeutic target for the cure of liver cancer. This study is the first to systematically evaluate the association of lncRNA, the expression quantity, and the clinical attributes and prognostic value in liver cancer patients, providing a basis for clinical practice.

## 2. Materials and Methods

### 2.1. Literature Search Strategy

We searched computers for EMBASE, PubMed, Web of Science databases, and the Cochrane Library to collect studies related to the correlation between high expression of lncRNA and prognosis of hepatic carcinoma. Only articles in English were selected. The following keywords were used: lncRNA, long ncRNA, lincRNAs, long noncoding RNA, long noncoding RNA, long untranslated RNA, liver neoplasm, hepatic neoplasm, hepatocellular cancer, liver cancer, cancer of the liver, etc. At the same time, manually search for references as a supplement.

### 2.2. Inclusion and Exclusion Standard

The standard for eligible articles is mentioned as (1) the case-control studies related to the correlation between high levels of lncRNA and prognosis of patients with hepatic carcinoma were published at home and abroad. (2) The affected individuals were diagnosed with hepatic carcinoma by cytological and histopathological examination. (3) The expression of lncRNA was quantified by reverse transcription-polymerase chain reaction (RT-PCR). (4) The cutoff value of lncRNA expression level was described. (5) Every study performed the association between expression of lncRNA and OS, and the hazard ratio (HR) value and its corresponding 95% confidence interval (95% CI) for OS was either obtained directly from actual study or indirectly it will be calculated by Engauge Digitizer 4.1 software from survival curve. (6) No restrictions of age, race, gender, and region.

The study exclusion standard is as follows: (1) repetitive published literature; (2) non-Chinese and English literature; (3) literature is unable to obtain full-text; (4) literature that does not report liver cancer prognosis outcomes or that cannot extract ending data from the text.

### 2.3. Data Extraction

Two researchers independently screen literature and extract data. Third researcher will handle if any disagreement occurs. Data was gathered and extracted based on the following criteria: (1) the basic information includes the topic of the study, author, and publication year; (2) baseline features of the included article, which included sample size, region, lncRNA type, lncRNA expression level, whether preoperative treatment, a cutoff value, lncRNA test method and TNM staging of liver cancer, etc. (3) Outcome indicators: OS, RFS, DFS, TNM stage, histological grade, vascular invasion, tumor numbers, tumor size, location, etc. The hazard ratio (HR) value and its corresponding 95% confidence interval (95% CI) for the OS, RFS, and DFS were either directly acquired from the original text or will be indirectly estimated by Engauge Digitizer 4.1 software from the survival curve [13]; (4) risk of bias assessed the key factors.

### 2.4. Quality Assessment of Included Studies

All the included studies were nonrandomized and retrospective studies. The quality was assessed using the Newcastle–Ottawa Scale (NOS). Each included study was assessed by two researchers for the quality from three mentioned items: “selection,” “comparability,” and “exposure.” There are evaluation items under each item, and each item is indicated by  when appropriate. The highest score of comparability is 2. Any discrepancies were resolved by consensus.

### 2.5. Statistical Analysis

We use Stata 16.0 software to perform statistical analysis. *P* < 0.01 was considered statistically significant. The odds ratio (OR) and hazard ratio (HR) were used to analyze the effect statistics, and each effect provided a 95% CI. Heterogeneousness between the comprised studies was analyzed using the *I*^2^ test. *I*^2^ ＜50% suggests no statistical heterogeneity between the outcomes of each research, using the fixed-effects model to perform the meta-analysis. Otherwise, the random-effect model would be used finally. After excluding the significant effects of clinical heterogeneity, use the random-effects model to perform the meta-analysis. Significant clinical heterogeneity is processed using methods such as subgroup analysis or sensitivity analysis [14].

## 3. Results

### 3.1. Literature Screening Process and Results

Overall, 4140 articles were retrieved in the early inspection. Later on, forty-two studies were finally included on layer-by-layer screening.  Figure 1 shows the literature screening process and outcomes.

### 3.2. Basic Characteristics and Quality Assessment Results of the Included Studies

General characteristics of liver cancer patients include age, gender, sample size, region, lncRNA type, lncRNA expression level, whether preoperative treatment, a cutoff value, etc. These all are shown in Table 1.

Newcastle–Ottawa Scale (NOS) marked included studies to be of high quality. All the studies have a score greater than 5 stars and meet the criteria for inclusion in the meta-analysis. The results are listed in Table 2.

### 3.3. Meta-Analysis Results

#### 3.3.1. Clinical Features

A total of 42 studies were included, including 6293 samples. Meta-analysis showed that patients with high expression of lncRNA had later TNM stage (OR = 0.36, 95%CI (0.31, 0.41), *P* < 0.001), lower histological grade (OR = 0.56, 95%CI (0.49, 0.65), *P* < 0.001), more vascular invasion (OR = 2.02, 95%CI (1.74, 2.35), *P* < 0.001), bigger tumor size (OR = 2.28, 95%CI (2.00, 2.60), *P* < 0.001), more severe liver cirrhosis (OR = 1.39, 95%CI (0.1.16, 1.66), *P* < 0.001), more likely to metastasize (OR = 1.80, 95%CI (1.49, 2.18), *P* < 0.001), more expression of AFP (OR = 1.46, 95%CI (1.22, 1.75), *P* < 0.001 and OR = 1.79, 95%CI (1.40, 2.29), *P* < 0.001), and more tumor numbers (OR = 0.72, 95%CI (0.62, 0.84), *P* < 0.05). The differences of other clinical features, such as age, gender, and HBV infection were not statistically significant. The results are shown in Table 3.

#### 3.3.2. OS

A total of 29 studies were included. The meta-analysis of the fixed effects model (I^2^ = 0.0%, *P* = 0.829) showed that compared with patients with low expression of lncRNA, patients of high expression of lncRNA have shorter OS. The difference was statistically significant (HR = 2.32, 95 CI% (2.08, 2.59), *P* < 0.01) (Figure 2).

#### 3.3.3. RFS

A total of 4 studies [21, 24, 30, 54] were included. The meta-analysis of the fixed effects model (I^2^ = 0.0%, *P* = 0.576) showed that compared with patients with low expression of lncRNA, patients with high expression of lncRNA have shorter RFS. The difference was statistically significant (HR = 2.19, 95 CI% (1.72, 2.78), *P* < 0.01) (Figure 3).

#### 3.3.4. DFS

A total of 7 studies [16, 20, 29, 31, 33, 41, 52] were included. The meta-analysis of the fixed effects model (I^2^ = 38.1%, *P* = 0.138) showed that compared with patients with low expression of lncRNA, patients with high expression of lncRNA have shorter DFS. The difference was statistically significant (HR = 2.01, 95 CI% (1.57, 2.57), *P* < 0.01) Figure 4.

## 4. Discussion

Liver cancer has a very powerful, invasive, and aggressive ability, and it is prone to distant metastasis and recurrence, which leads to extremely mortality rate. In China, most patients with liver cancer are in an advanced stage when they are diagnosed, and the treatment methods and the effects are fantastically limited for them. Hence, the initial diagnosis and treatment of hepatic carcinoma remains a global difficulty and generates a large amount of discussion. Although there is an ongoing emergence of new drugs and treatments for liver cancer, there remain many difficulties in the early diagnosis and postoperative prognosis. Thus, the development of novel effective molecular therapeutic targets is the need of time to enhance the rate of diagnosis rate of liver cancer and the accuracy of prognosis judgment [56]. In recent years, according to detecting the tissues and plasma of cancer patients by real-time reverse transcription-polymerase chain reaction (RT-PCR), a high quantity of aberrantly expressed lncRNAs is found to participate in tumor metabolism to promote tumor development in different ways [57]. It has been found that only 1.5% of nucleic acid sequences were coding that is they make proteins while the rest 98.5% of the sequences are noncoding RNAs in three billion base pairs of the human genome, the latter regulated gene expression and maintained intracellular homeostasis through chromosome alteration, regulation of transcription, and posttranscriptional regulation. LncRNA dysregulation can cause chromosome loss and translocation, leading to the occurrence of cancer [58, 59]. Thus, lncRNA may be a potential biological target or as a molecular drug for prognosis and early diagnostic screening of cancer. At present, the relationship between lncRNA and tumor is attracting worldwide attention. Wang et al. [60] identified PVT1 to be highly expressed in hepatocellular carcinoma and related cell lines, and the affected individuals with increased PVT1 expression have a poor prognosis. PVT1 can increase the stability of nuclear protein NOP2, which helps cell proliferation, tumorigenesis, and gaining the same characteristics as exhibited by stem cells. Li et al. [61] found significantly increased HOTAIR expression level in liver cancerous tissues than paracarcinoma tissue. Besides, HOTAIR could downregulate the expression and phosphorylation of SETD2 to inhibit repair of DNA damage, causing microsatellite variability and aberrant cell cycle-related gene expression, which could further promote the occurrence of liver cancer. Yang [62] reported a crucially high expression level of noncoding RNA HEIH in affected individuals as compared to healthy ones. With the increase of the TNM stage, the expression of plasma HEIH increased gradually. LAN [63] found SNHG12 to be increasingly expressed in liver cancer-specific individuals and are connected with cancer size, TNM stage, and vascular invasion. Affected individuals with increased expression of SNHG12 had a worse prognosis and a higher recurrence rate than patients with low expression. SNHG12 can adsorb miR-199a/b-5p to increase the expression of MLK3 and its downstream effector molecule in the NF-*κ*B pathway. Wang [64] reported that CARLo-5 is highly expressed in HCCLM3 and MHCC97-L cell lines and promotes the proliferation and metastasis of HCC, causing threats to the general and disease-free survival of affected individuals. These outcomes suggest that different types of lncRNA play different characters, but they all have significant roles in the growth and prognosis of liver cancer. Consequently, if one or more specific lncRNAs related to liver cancer are screened, chip technology, real-time quantitative RT-PCR, in situ hybridization technique, and other technologies can help in measuring the expression level of patients' blood, urine, and other body fluids during clinical diagnosis and treatment, thereby improving the early diagnosis and prognosis of liver cancer.

The present work is the first one to analytically evaluate the relationship between the expression level of lncRNA and the clinical features and prognostic rate of affected individuals. The results show that vascular invasion, histological grade, number of tumors, size of the tumor, metastasis, and TNM stage of liver cancer patients are associated with the expression level of lncRNA. Furthermore, the patients with high expression of lncRNA have shorter OS, RFS, and DFS than those with low expression. The above results have statistically significant values, and the heterogeneity is very weak. So, the high expression of lncRNA may be a reason for decreased prognosis of hepatic carcinoma. But so far, the research on lncRNA is still in the preliminary stage. Currently, only a few lncRNAs are found, but there are still a high number of purposes and regulatory mechanisms of lncRNAs which are not clear. Moreover, these lncRNAs related to liver cancer have been confirmed by previous studies, but its clinical application in tumor diagnosis and treatment remain to be further explored. lncRNA has a good prospect of diagnosis and treatment, and it can become a new star of tumor marker in the future, providing new hope for the targeted therapeutic of hepatic carcinoma and the development of anticancer drugs.

Limitations of present work: (1) the comprised studies were retrospective studies, and the study design may have the risk of recall, measurement, and reporting bias; (2) the comprised research studies were all from China, due to differences in etiology, pathology, and prognosis in different regions. Therefore, this conclusion cannot be extended to other regions; (3) HRs of some included studies are not directly given relevant outcome indicators and only manually retrieved from the survival curve and then calculated, which may influence the validity of the results.

In conclusion, the highest expression of lncRNA in liver cancer patients is a poor prognosis factor for liver cancer. Owing to the limitations of the quantity and quality of researchers involved, the above deductions are subject to verification by further studies.

## Figures and Tables

**Figure 1:** The flow chart of literature screening process.

**Figure 2:** Forest plots for the relationship between the overexpressed lncRNA and OS. The center of each square represents the HR, the area of the square is the number of sample and the weight used in the meta-analysis, and the horizontal line indicates the 95%CI. CI indicates confidence interval; HR: hazard ratio.

**Figure 3:** Forest plots for the relationship between the overexpressed lncRNA and RFS. RFS indicates recurrence-free survival.

**Figure 4:** Forest plots for the relationship between the overexpressed lncRNA and DFS. RFS indicates disease-free survival.

**Table 1:** Basic characteristics of included studies.

Study ID	Region	Sample Size	lncRNA	Cutoff Value	TNM Stage	Data extraction method	Follow-up (months)	Outcome	Postoperative treatment
Guo [15]	China	95	NEAT1	Median value	I–IV	Survival curve	No	OS	NO
Hua [10]	China	92	ANRIL	Median value	I–IV	Reported in text	60	OS	NO
Li [16]	China	179	GHET1	Median value	I–IV	Reported in text	No	OS + DFS	NO
Wang [17]	China	112	HOXA-AS2	Median value	I–IV	Survival curve	No	OS	NO
Zhou [18]	China	109	BANCR	Median value	I–III	Survival curve	SDD	OS	NO
Ding [19]	China	137	TUG1	Median value	I–IV	Reported in text	No	OS	NO
Ding [20]	China	214	PVT1	ROC analysis	I–IV	Reported in text	27.58	OS + RFS	NR
Yang [21]	China	60	HOTAIR	ROC analysis	—	Reported in text	18.6	OS + RFS	NR
Yan [22]	China	117	PCAT-1	Median ratio	—	Reported in text	60	OS	NO
Zhang [23]	China	144	SNHG3	Median value	I–IV	Reported in text	60	OS	NO
Dong [24]	China	84	PlncRNA-1	Median value	I–IV	Both	No	OS + RFS	NR
Shi [25]	China	84	Sox2ot	Median ratio	I–IV	Reported in text	60	OS	NO
Li [26]^50^	China	102	ZEB1-AS1	Median value	I–III	Survival curve	SDD	OS	NO
Shen [27]	China	100	SNHG7	Mean ratio	I–IV	Both	84	OS	NR
Zhang [28]	China	55	UCA1	Median value	I–IV	Both	60	OS	NO
Zhang [29]	China	127	RHPN1-AS1	median value	I–IV	Both	60	OS + DFS	NO
Jiao [30]	China	370	SNHG4	ROC analysis	I–IV	Reported in text	No	OS + RFS	NO
Xiao [31]	China	100	GIHCG	ROC analysis	I–IV	Reported in text	60	OS + DFS	NR
Zhang [32]	China	337	ROR1-AS1	Mean ratio	I–IV	Reported in text	No	OS	NR
Zeng [53]	China	130	CASC9	Median value	I–IV	Reported in text	60	OS	NR
Bai [54]	China	353	PTTG3P	Youden index	I–IV	Reported in text	72	OS + RFS	NO
Nie [33]	China	371	ACVR2B-AS1	—	I–IV	Reported in text	No	OS + DFS	NO
Fu [34]	China	122	CCAT2	Median value	I–IV	Reported in text	60	OS	NR
Zhao [35]	China	161	ENST00000429227.1	—	—	Reported in text	No	OS	NO
Pan [36]	China	59	circ0000267	Median value	I–IV	Reported in text	60	OS	NO
Zhong [55]	China	108	SNHG16	Median value	—	Reported in text	60	OS	NR
Wang [37]	China	127	LINC0051 1	Median value	I–IV	Reported in text	60	OS	NR
Guo [38]	China	61	SNGH16	Positive evels	I–IV	Reported in text	60	OS	NR
Wang [39]	China	101	MIR210HG	Median value	I–IV	Both	120	OS + DFS	NR
Wang [40]	China	40	LINC01296	—	I–IV	Survival curve	No	OS	NR
Zhou [41]	China	197	HOXC13-AS	median value	I–IV	Reported in text	60	OS + DFS	NO
Yu [42]	China	123	SUMO1P3	Median value	I–IV	Reported in text	60	OS	NR
Huang [43]	China	136	PTTG3P	—	I–IV	Reported in text	60	OS	NR
Tang [44]	China	66	RUSC1ASN	—	—	Survival curve	72	OS + RFS	NR
Qi [45]	China	70	lncPARP1	—	—	Survival curve	36	OS + DFS	NO
Jin [46]	China	161	MINCR	—	I–IV	Reported in text	60	OS	NO
Xu [47]	China	108	TRPM2-AS	Normal value	—	Survival curve	72	OS	NO
Li [48]	China	193	AK021443	Mean ratio	I–IV	Reported in text	No	OS	NO
Li [49]	China	68	GHET1	Mean ratio	—	Survival curve	60	OS	NO
Wang [50]	China	326	LRB1	Median value	I–IV	Survival curve	72	OS	NR
Zeng [51]	China	84	LncDQ	—	I–IV	Reported in text	60	OS	NR

*Note.* Cutoff value: the critical value to distinguish between high and low lncRNA expression; OS : overall survival; mean ratio: average expression level of lncRNA; median value: median expression level of LncRNA; — : no mention in text; OS : overall survival; DFS : disease-free survival; RFS : relapse-free survival; both: reported in text and survival curve; SDD : surgery to the date of death.

**Table 2:** The quality evaluation results of included studies by NOS.

Study ID	Selection	Comparability	Outcome	Score
Yang [21]	★★	★★	★★★	7
Guo [15]	★★	★★	★★★	7
Hua [10]	★★	★★	★★	6
Ding [20]	★★	★★	★★★	7
Yan [22]	★★	★★	★★★	7
Shi [25]	★★	★★	★★★	7
Wang [17]	★★	★★	★★★	7
Zhou [18]	★★	★★	★★★	7
Zhang [23]	★★★	★★	★★★	8
Dong [24]	★★	★★	★★★	7
Li [26]	★★	★★	★★	6
Li [16]	★★	★★	★★★	7
Ding [19]	★★	★★	★★★	7
Huang [43]	★★	★★	★★★	7
Tang [44]	★★	★★	★★★	7
Qi [45]	★★	★★	★★★	7
Jin [46]	★★	★★	★★★	7
Xu [47]	★★	★★	★★	6
Li [48]	★★	★★	★★★	7
Li [49]	★★	★★	★★★	7
Wang [50]	★★	★★	★★★	7
Zeng [51]	★★★	★★	★★★	8
Zhang [32]	★★★	★★	★★	7
Zeng [53]	★★	★★	★★★	7
Bai [54]	★★★	★★	★★★	8
Nie [33]	★★	★★	★★	6
Fu [34]	★★	★★	★★★	7
Zhao [35]	★★	★★	★★	6
Pan [36]	★★	★★	★★★	7
Zhong [55]	★★	★★	★★	6
Wang [37]	★★	★★	★★★	7
Guo [38]	★★	★★	★★★	7
Wang [39]	★★	★★	★★★	7
Wang [40]	★★	★★	★★★	7
Zhou [41]	★★	★★	★★★	7
Shen [27]	★★	★★	★★★	7
Zhang [28]	★★	★★	★★★	7
Zhang [29]	★★	★★	★★★	7
Zhang [5]	★★★	★★	★★	7
Jiao [30]	★★★	★★	★★	7
Xiao [31]	★★★	★★	★★★	8
Yu [42]	★★	★★	★★★	7
Liang [52]	★★	★★	★★★	7

**Table 3:** Results of meta-analysis on the correlation between LncRNA expression level and clinical features of liver cancer.

Clinical Characteristics	Number of studies included (papers)	Tests for heterogeneity		Effect of the model	Results of meta-analysis	
		*I* ^2^ (%)	*P* value		OR (95%CI)	*P* value
Age	39 [5, 10, 16–52]	66.5%	<0.001	Random	1.07 (0.96, 1.19)	0.253
Gender	42 [5, 10, 16–55]	0.0%	0.66	Fixed	1.03 (0.92,1.15)	0.648
Tumor size	33 [10, 16, 29, 31, 34, 36, 39, 41–52]	71.8%	<0.001	Random	2.28 (2.00,2.60)	<0.001
HBV infection	25 [10, 16, 19, 20, 24, 25, 27, 29, 31, 34, 36, 39, 41, 43, 44, 46, 52, 55]	0.0%	0.712	Fixed	1.12 (0.95,1.31)	0.182
Liver cirrhosis	18 [16, 20, 22, 25, 34, 38, 42, 44, 47, 49, 51, 55]	0.0%	0.799	Fixed	1.39 (1.16,1.66)	<0.001
Metastasis	16 [22, 23, 27, 28, 30, 34, 37, 38, 40, 41, 48, 51, 52]	72.5%	<0.001	Random	1.80 (1.49,2.18)	<0.001
H- grade	28 [5, 10, 16, 25, 28, 30, 32, 33, 35, 37, 39, 41, 42, 45, 48, 53, 54]	67.5%	<0.001	Random	0.54 (0.48,0.62)	<0.001
AFP (400)	18 [10, 16, 22, 24, 26, 35, 36, 41, 45, 47, 51, 52, 55]	41.5%	0.034	Fixed	1.46 (1.22,1.75)	<0.001
AFP (20)	9 [27, 29, 40, 42, 43, 46, 48, 50]	76.9%	<0.001	Random	1.79 (1.40,2.29)	<0.001
TNM stage	33 [5, 10, 15, 20, 22, 24, 34, 36, 43, 46, 48, 50, 51, 54]	78.9%	<0.001	Random	0.46 (0.41,0.51)	<0.001
Tumor number	25 [10, 16, 24, 26, 29, 31, 34, 35, 37, 42, 43, 46, 48, 50, 51, 55]	53.4%	0.001	Random	0.72 (0.62,0.84)	<0.001
V-invasion	22 [16, 19, 24, 26, 30, 32, 35, 37, 41, 42, 44, 45, 47, 49, 51, 55]	84.7%	<0.001	Random	2.02 (1.74,2.35)	<0.001

AFP (400): the cutoff of AFP is 400 *μ*g/L; AFP (20): the cutoff of AFP is 20 *μ*g/L; *H*-grade: histological grade; *V*-invasion: vascular invasion.

## Data Availability

The data could be obtained from contacting corresponding author.

## Abbreviations

RNA: Ribonucleic acid
lncRNA: Long noncoding RNA
TNM: Tumor, node, metastasis
OR: Odds ratio
95%CI: 95% confidence interval
ORF: Open reading frame
RT-PCR: Reverse transcription-polymerase chain reaction
OS: Overall survival
DFS: Disease-free survival
RFS: Relapse-free survival
HR: Hazard ratio
NOS: Newcastle–Ottawa Scale
PVT1: Plasmacytoma variant translocation 1
NOP2: Nucleolar protein 2
HOTAIR: HOX transcript antisense RNA
SETD2: SET domain containing 2.
